The article "Modified Lamaze Breathing Reduces Abdominal Pain in Patients during Colonoscopy" was retracted in 2023. Reasons: signs of a paper mill; suspected computer-generated content; unreliable results or conclusions; concerns about the data.

# Modified Lamaze Breathing Reduces Abdominal Pain in Patients during Colonoscopy

**DOI:** 10.1155/2022/1557861

**Published:** 2022-07-26

**Authors:** Fuqun Wang, Shizhen Wen, Jing Chen, Liwen Du, Juncheng Zeng

**Affiliations:** ^1^Department of Gastroenterology, Meizhou People's Hospital, Meizhou 514000, China; ^2^Digestive Endoscopy Center, Meizhou People's Hospital, Meizhou 514000, China

## Abstract

**Objective:**

To study the effects of modified Lamaze breathing on abdominal pain experienced during colonoscopy.

**Methods:**

Eighty-five patients who underwent common colonoscopy at our hospital between March 2021 and May 2021 were selected and randomly divided into the Lamaze group (*n* = 40) and a control group (*n* = 45). Their basic clinical information was collected, and the bowel cleanliness, the time for the endoscope to reach the ileocecal junction, and the degree of abdominal pain of the two groups were compared.

**Results:**

No significant difference was observed in age, gender, bowel cleanliness, and time of endoscope to reach the ileocecal junction between the two groups. However, the degree of abdominal pain (anal region, descending sigmoid colon junction, splenic flexure, and hepatic flexure) was significantly lower in the Lamaze group compared with the control group.

**Conclusion:**

Modified Lamaze breathing demonstrated promising effectiveness in reducing abdominal pain during colonoscopy and improving the quality of the examination.

## 1. Introduction

Colonoscopy, despite being a modern minimally invasive procedure with high accuracy in diagnosing colorectal diseases [1], may still trigger symptoms such as abdominal pains, abdominal distension, elevated blood pressure, and increased heart rate during examination [2–4]. Some patients may also suffer from shortness of breath, leading to respiratory alkalosis with manifestations such as numbness and convulsions of lips, cheeks, and fingers, and an increased incidence of abdominal pain and tissue injury [5]. Although anesthesia and analgesia can improve colonoscopy-associated pain in patients, they may be unsuitable for many patients due to other attributable risks of anesthesia, postoperative care, and costs [6]. Therefore, there is an urgent need to find appropriate adjuvant methods to combine with colonoscopy procedures to relieve patients' pain.

Lamaze breathing originates from the “Lamaze method of childbirth,” first developed by French obstetrician Ferdinand Lamaze [7]. It is an intervention method that was shown to reduce pain by regulating breathing and allowing parturients to actively control pain and other discomforts caused by contractions during delivery via structured breathing and muscle relaxation [8, 9]. Lamaze breathing is widely used during spontaneous delivery of parturients due to its ability to effectively shift the women's attention during delivery and relieve muscle pain and stress.

The article "Modified Lamaze Breathing Reduces Abdominal Pain in Patients during Colonoscopy" was retracted in 2023. Reasons: signs of a paper mill; suspected computer-generated content; unreliable results or conclusions; concerns about the data.

During a colonoscopy, the colon is stretched after a gas injection, which may cause pain and discomfort in the patients. The mechanisms of labor pain and colonoscopy-caused pain may be similar to a certain extent since the colon and uterus contain smooth muscles [10].

In this study, we made patients undergoing colonoscopy to perform a modified Lamaze breathing technique and assessed its effects on the degree of abdominal pain to provide a new research direction for improving the quality of clinical enteroscopy.

## 2. Materials and Methods

### 2.1. Study Subjects

The data of 85 patients who underwent colonoscopy at the Digestive Endoscopy Center of our hospital between March 2021 and May 2021 were collected and randomly classified into the Lamaze group (*n* = 40) and control group (*n* = 45). In the control group, routine nursing interventions for colonoscopy were performed, while for the Lamaze group, modified Lamaze breathing was performed in addition to routine nursing interventions.

Inclusion criteria of participants were as follows [10]: (1) normal cognitive and communication ability; (2) ability to understand and complete the questionnaire; (3) willingness to perform the “modified Lamaze breathing” during colonoscopy; and (4) providing informed consent. The study exclusion criteria were as follows: (1) severe cardiovascular and respiratory diseases; (2) history of abdominal/pelvic surgery or inflammatory bowel disease; (3) complete blindness, severe visual impairment, deaf-mutism, inability to read, listen, watch, or understand written, voice, or video materials; (4) severe mental illness or cognitive impairment; (5) inability to communicate normally due to other reasons; (4) inability to move freely in bed; and (6) recent acute lower gastrointestinal bleeding. The general data of the patients was recorded. Informed consent was obtained from all patients. This study was approved by the Ethics Committee of Meizhou People's Hospital (2021-C-55).

### 2.2. Modified Lamaze Breathing Method of Colonoscopy

This technique was performed based on the following steps:

Step A: thoracic breathing at the beginning of the examination: (1) complete relaxation; (2) staring at one point; (3) inhaling through the nostrils and exhaling through the mouth, with the abdomen relaxed; and (4) 6-9 times of inspiration and exhalation per minute

Step B: shallow and slow accelerated breathing when the colonoscopy passed through the descending sigmoid colon junction (mild pain): (1) complete relaxation; (2) staring at one point; (3) inhaling through the nostrils and exhaling through the mouth; and (4) accelerating breathing with increasing pain and slowing it down with decreasing pain

Step C: shallow breathing when the colonoscopy passed through the splenic flexure and hepatic flexure (pain above moderate degree): (1) complete relaxation; (2) staring at one point; (3) exhaling with a slightly opened mouth (emitting “hee hee” sounds), making noise from the larynx; (4) adjusting respiratory rate according to the intensity of pain, with the amount of air inhaled and exhaled kept the same to avoid hyperventilation; and (5) 4-6 continuous rapid breaths followed by forced exhalation. This step was repeated until the pain disappeared

Step D: halitus movement when feeling pain but unable to gather strength: to open the mouth and breathe rapidly like gasping with the body relaxed

The article "Modified Lamaze Breathing Reduces Abdominal Pain in Patients during Colonoscopy" was retracted in 2023. Reasons: signs of a paper mill; suspected computer-generated content; unreliable results or conclusions; concerns about the data.

### 2.3. Evaluation of Bowel Cleanliness [10]

All examined patients took the same laxative for bowel preparation, and the quality of preparation was graded as follows: grade I, excellent with no visible feces; grade II, satisfactory with a small amount of visible feces, but did not block the visual field; and grade III, unsatisfactory with feces blocking the visual field and/or colonoscopy passage.

### 2.4. Pain Assessment

After the colonoscopy, the patients' intraoperative pain was measured with the Wong-Baker faces pain rating scale [11]. Patients were advised to score their degree of pain during the examination using the Wong-Baker faces pain rating scale. A score of 0 indicated no pain, 2 indicated hurts a little bit, 4 indicated hurts a little more, 6 indicated hurts even more, and 10 indicated hurts worst.

### 2.5. Statistical Analysis

The SPSS 24.0 software was used for data analysis. Measurement data were expressed as mean ± standard deviation (SD), and the *t*-test was used for comparison between the two groups and Wilcoxon rank-sum test for nonnormal distribution variables. Enumeration data were expressed as frequency (*n*) and percentage (%), and the chi-square test was used for statistical analysis. *P* < 0.05 was considered statistically significant.

## 3. Results

### 3.1. General Information of Patients

The general data of the patients included were analyzed. According to the results, there were no significant differences between the Lamaze group and control group in terms of gender, age, and history of colonoscopy (Table 1), indicating that the two groups of patients were comparable, and there was no previous history of abdominal surgery in either group, and no complications occurred after microscopy.

The article "Modified Lamaze Breathing Reduces Abdominal Pain in Patients during Colonoscopy" was retracted in 2023. Reasons: signs of a paper mill; suspected computer-generated content; unreliable results or conclusions; concerns about the data.

### 3.2. Comparison of Bowel Cleanliness between the Two Groups

Bowel preparation was evaluated in both groups of patients during colonoscopy. The results showed that the intestinal tract of patients in both groups was clean without stool accumulation; there was no significant difference in bowel cleanliness between the two groups (Table 2), indicating that the degree of pain during colonoscopy was comparable between the two groups.

### 3.3. Comparison of the Time of Endoscope Reaching the Ileocecal Junction between the Two Groups

The duration of colonoscopy was compared between the two groups. It was revealed that there was no significant difference in the time to reach the ileocecal junction between the two groups (Table 3).

### 3.4. Comparison of Abdominal Pain during Colonoscopy between the Two Groups

The degree of abdominal pain caused during colonoscopy was compared between the two groups. The results showed that patients in the control group experienced significantly more intense pain in the anal region, descending sigmoid colon junction, splenic flexure, and hepatic flexure than those in the Lamaze group (Table 4), suggesting that the modified Lamaze breathing could effectively relieve abdominal pains in patients during colonoscopy.

## 4. Discussion

Colonoscopy, as the main means of examination for colorectal diseases worldwide, is of great value for the early detection of colorectal lesions [12]. However, many difficulties must be overcome for colonoscopy to be accepted by patients due to various degrees of abdominal pain triggered by the insertion of an endoscope and repeated injection of air into the enteric cavity [13]. In recent years, sedative colonoscopy has been rapidly developed, improving patients' willingness to undergo colonoscopy [11, 14], but some complications associated with colonoscopies such as bleeding, gastric perforation, and cardiopulmonary injury persist [15]. Some scholars have also reported some nonsedative colonoscopies, such as music and warm water infusion [16, 17], which, however, have not been widely used and promoted due to certain limitations. Lamaze breathing is an effective pain-relieving method applied during delivery, also known as psychoprophylactic preparation for childbirth [18]. Parturients are equipped with Lamaze breathing techniques before delivery, effectively shifting their attention to breathing control, resulting in less focus on pain and allowing moderate relaxation of muscles [19].

The pain arising from colonoscopy falls into the category of visceral pain, often caused by stimuli such as mechanical traction, intestinal smooth muscle spasm, ischemia, and inflammation, leading to unpleasant feelings accompanied by nausea, vomiting, and changes in cardiovascular and respiratory activities. As reported, to provide an effective field of view during colonoscopy, air injection is required to dilate the intestinal cavity, but excessive air can cause the intestinal lumen to be overinflated and stretched, stimulating nerve endings to produce pain. Since the colon is relatively free in the abdominal cavity, abdominal pain, abdominal distension, nausea, and vomiting can be triggered when the endoscope passes through bends such as the descending sigmoid colon junction, hepatic flexure, and splenic flexure. When the bowel is stimulated during colonoscopy, smooth muscle spasm of the bowel wall can occur, thus producing pain [20], similar to the mechanism of pain during delivery. Lamaze breathing can help maintain a relatively constant position of the intestine by deepening abdominal breathing, making the colonoscope easy to pass through and producing pain relief.

The article "Modified Lamaze Breathing Reduces Abdominal Pain in Patients during Colonoscopy" was retracted in 2023. Reasons: signs of a paper mill; suspected computer-generated content; unreliable results or conclusions; concerns about the data.

In this study, the pain-relieving effects of modified Lamaze breathing during colonoscopy were observed due to the advantages of Lamaze breathing and the characteristics of colonoscopy. The study results showed that there was no significant difference in age, gender, colonoscopy history, occurrence of complications, and time of the endoscope to reach the ileocecal junction between the two groups. Compared with routine nurse interventions for colonoscopy, Lamaze colonoscopy could significantly reduce the pain score of anal pain, descending sigmoid colon junction, splenic flexure, and hepatic flexure, which was consistent with findings of Yu et al. and T. Voiosu et al. [10, 21].

Bowel cleanliness is also associated with the degree of abdominal pain in patients. Fecal water and bubbles in the enteric cavity can directly affect endoscopists' visual field, increasing the risk of missed diagnosis and treatment difficulties. Multiple repeated irrigation will increase the operation time and cause discomfort. Thus, poor intestinal cleanliness leads to more time for endoscopists to intubate, which could result in a higher rate of failure [22]. However, in this study, no significant differences were observed in the degree of bowel cleanliness between the two groups of patients, which may be attributed to the presence of more success factors for examination.

## 5. Conclusions

Performing modified Lamaze breathing preoperatively under proper guidance could subdue abdominal pain during colonoscopy, increase patients' tolerance, and enhance their experience during medical treatment.

## Figures and Tables

**Table 1:** General data of the included patients.

Variables	Lamaze group (n =40)	Control group (n =45)	*χ* ^2^/T	*P*
Gender			0.93	0.34
Male	28	27		
Female	12	18		
Age (years)	48.28 ± 12.74	47.87 ± 14.32	0.14	0.89
History of colonoscopy			0.51	0.47
Yes	13	18		
No	27	27		

The article "Modified Lamaze Breathing Reduces Abdominal Pain in Patients during Colonoscopy" was retracted in 2023. Reasons: signs of a paper mill; suspected computer-generated content; unreliable results or conclusions; concerns about the data.

**Table 2:** Comparison of bowel cleanness between the two groups.

Group	Cases (*n*)	Grade I	Grade II	Grade II-III	Grade III	*Z*	*P*
Lamaze group	40	13	22	2	3		
Control group	45	14	27	2	2	0.1199	0.9046
Total	85	27	49	4	5		

Note: using the rank-sum test, *P* > 0.05 indicated no significant difference in bowel cleanliness.

**Table 3:** Comparison of time of endoscope reaching the ileocecal junction between the two groups (min).

Group	Cases (*n*)	Mean	Median	Minimum	Maximum	*P*
Lamaze group	40	5.13	5	1	10	0.2027
Control group	45	6.36	5	2	40	
Total	85	5.78	5	1	25	

**Table 4:** Comparison of abdominal pain between the two groups.

Group	Cases (*n*)	Wong-Baker faces pain rating scale (points)					*Z*	*P*
		0	2	4	6	8		
Pain assessment in the anal region								
Lamaze group	40	39	1	0	0	0		
Control group	45	35	10	0	0	0	2.6879	0.0072^∗∗^
Total	85	74	6	0	0	0		
Pain assessment in the descending sigmoid colon junction								
Lamaze group	40	21	17	1	1	0		
Control group	45	1	17	20	6	1	6.1017	<0.0001^∗∗∗^
Total	85	22	34	21	7	1		
Pain assessment in the splenic flexure								
Lamaze group	40	17	18	4	1	0		
Control group	45	1	8	19	15	2	6.2996	<0.0001^∗∗∗^
Total	85	18	26	23	16	2		
Pain assessment in hepatic flexure								
Lamaze group	40	15	16	6	3	0		
Control group	45	0	12	16	14	3	5.2493	<0.0001^∗∗∗^
Total	85	15	28	22	17	3		

Note: ^∗∗^*P* < 0.01 and ^∗∗∗^*P* < 0.001 vs. control group.

## Data Availability

The data used to support the findings of this study are available from the corresponding author upon request.
